The article "Pathological dislocation of the hip due to coxotuberculosis in children: a 29-case report" was retracted in 2015. Reason: compromised peer review.

# Pathological dislocation of the hip due to coxotuberculosis in children: a 29-case report

**DOI:** 10.1186/1749-799X-9-16

**Published:** 2014-03-10

**Authors:** Xin Jiang, Yuan Li, Lijun Liu, MingXin Peng, XueYang Tang, DaoXi Wang, XiaoDong Yang

**Affiliations:** 1 Department of Pediatric Surgery, West China Hospital, Sichuan University, No. 37 Guoxue Road, Chengdu, Sichuan 610041, People's Republic of China

**Keywords:** Pathological hip dislocation, Coxotuberculosis, Open reduction, Acetabular reconstruction

## Abstract

**Background:**

The aim of this study is to evaluate the clinical outcome of various surgery methods in children suffering pathological dislocation of the hip joint due to coxotuberculosis.

**Patients and methods:**

From January 2006 to January 2011, 29 children with coxotuberculosis hip dislocation were treated with open reduction (4 children) and acetabular reconstruction (25 children). According to degree of dislocation and age, acetabular reconstructions included Salter osteotomy (nine children), Pemberton operation (six children), Dega operation (seven children), the hip shelf arthroplasty (two children), and Chiari operation (one child). During acetabular reconstruction, 16 children underwent upper femoral rotational shortening osteotomies simultaneously, 6 children underwent the femoral head and neck reconstruction simultaneously, and 3 children were underwent corrective osteotomy. After operation, children were immobilized with plaster external fixation for 1–3 months and treated with routine anti-infective therapy for 3 days. During follow-up study (12–18 months), the hip stability was examined via X-ray. The recovery was evaluated via acetabular index (AI) and Harris hip score.

**Results:**

Postoperative X-ray films of 29 children showed concentric reduction of all hips. Total 25 children healed I incision surgery, while 4 children with skin antrum of incision were further treated leading to 1–3 months delay of healing. Total 24 children were followed up for 2–5 years. X-ray examination revealed no redislocation after 2 years postoperative. The postoperative AI was normal (15°–20°) in 22 children and increased to 25°– 30° in 2 children. After 2 years postoperative, 8 children had normal function of hip joint, 13 children had mild limitation of flexion and rotation, and 3 children had fibrous ankylosis. The average of Harris hip score was 83 (ranged, 62–90).

**Conclusion:**

In our study, pathological hip dislocations of children attributed to coxotuberculosis were treated via open reduction and acetabular reconstruction and the outcomes were both excellent. Individual characteristic should be taken into consideration during treatment, and proper surgery approach should be adopted according to pathological changes of the hip.

The article "Pathological dislocation of the hip due to coxotuberculosis in children: a 29-case report" was retracted in 2015. Reason: compromised peer review.

## Introduction

Pathological dislocation of the hip joint in children is relatively rare occurrence and may cause lifelong disability when missed or ill-treated. The hip is a deep-seated articulation, and its dislocation may either remain hidden for some time or go undiagnosed [1]. According to the development of hip dislocation, pathological dislocation of the hip is frequently associated with heavy bone destructive defect of acetabulum and femoral heads and necks as well as the residual anatomic deformity. Therefore, this disease is difficult to treat, and several surgery operations have been explored and showed different outcomes.

Tuberculosis of the hip presents significant clinical problems, accounting for approximately 15% of osteoarticular tuberculosis [2]. The disease once occurred in the hip may lead to progressive destruction of the joint if untreated at an early stage, and many even proceed to pathological dislocation. Dislocated hips with infection are difficult to be managed to obtain a stable, mobile, congruous, and concentric joint. Diagnosis and effective treatment at an early stage are vital to treat the disease and save the joint [3]. The reports on the management of residual anatomic deformity of hip dislocation due to tuberculosis in children have rarely been documented. No comprehensive treatment protocol has been outlined.

From 2006 to 2011, we have performed surgery approaches in 29 children with pathological tubercular dislocation of the hip, accounting for 3.4% of hip dislocation in our hospital. The details of the patients' general data and clinical results are presented here.

## Patients and methods

This study was approved by the Institutional Review Board of West China Hospital, Sichuan, China. Written informed consent was obtained from the patients for the publication of this report and any accompanying images. Based on the diagnosis card index at our department during the period from January 2006 to January 2011, we searched the files of patients with pathological hip dislocation caused by tuberculosis. Patients were included in the study if they met the following criteria: no previous treatment in other hospitals and radiographs available from the start of treatment to healing. Patients with slight subluxation or acetabular dysplasia were excluded.

Clinical manifestation of 29 patients with hip dislocation due to coxotuberculosis was shown in Table 1. Total 29 children (13 boys and 16 girls) with an average age of 4.3 years (ranged, 1–11 years) were included in the present study. There were 12 Han Chinese, 9 ethnic Tibetans, and 8 Yi people. Pathological tubercular hip dislocation is located in the right hip (17 children) and left hip (12 children). Four children showed subluxation of the hip joint, and 25 showed total dislocation of the hip. The mean duration of hip dislocation was 18 month (ranged, 10 days to 10 years). Besides the hip pain and lameness, other accompanied symptoms included significant local swelling in hip (13 children), fever (38°C–39°C) (6 children), pulmonary tuberculosis (7 children), spinal tuberculosis (2 children), tibia tuberculosis (1 child), femoral tuberculosis (1 child), and iliac fossa abscess (1 child). The function status of injured hip joint was assessed using the Harris hip score [4,5]. The average of preoperative Harris hip score was 61 (ranged, 43–78). All children presented the increased erythrocyte sedimentation rate, and the PPD skin test was positive in 23 children. Preoperative X-ray examination was performed for all children, and other examinations included computed tomography (CT) scan and three-dimensional reconstruction (23 children), color Doppler ultrasound (18 children), and magnetic resonance imaging (MRI) (12 children). The radiologic examination indicated the hip dislocation in all patients accompanied by avascular necrosis of femoral head (15 children), excalation of femoral head (6 children), total absence of femoral head (2 children), and absence of femoral head and neck (1 child). Additionally, eight children had increased anteversion angle (40°–60°) and three had varus deformity. The acetabular index (AI) was measured according to Kleinberg and Lieberman [6] on the primary radiographs. It was roughly normal in 11 patients with the values of 15°–20° and increased to 25°–35° in 12 patients and to 40°–50° in 6 patients.

The article "Pathological dislocation of the hip due to coxotuberculosis in children: a 29-case report" was retracted in 2015. Reason: compromised peer review.

**Table 1:** Clinical manifestation of 29 patients with hip dislocation due to coxotuberculosis

**Clinical manifestation**	**Patients**
Patients **(male/female)**	32 (19/13)
Age **(years)**	4.3 (ranged, 1–11)
Han/Tibetan/Yi nationality	12/9/8
Duration **(months)**	18 (ranged, 10 days–10 years)
Dislocation of hip joint	
Subluxation	4
Complete dislocation	25
Concomitant symptom	
Hip local swelling	13
Fever (38°C–39°C)	6
Pulmonary tuberculosis	7
Spondylocace	2
Tibia tuberculosis	1
Femoral tuberculosis	1
Liac fossa abscess	1
Harris score	61 (43–78)
Acetabular index	
15-20° (normal)	11
25-35° (mild)	12
40-50° (severe)	6
Preoperative examination	
Damage of acetabulum	18
Ischemic necrosis of femoral head	15
Excalation of femoral head	6
Total absence of femoral head	2
Absence of femoral head and neck	1

### Surgical approaches

For the management of active tuberculosis of the hip, all patients were given routine antituberculosis therapy for 2–4 weeks before surgery. After routine preoperative preparations, patients were placed in a supine position and the contralateral hip was raised. Then, a Salter anterior approach to the hip was performed after intubation and general anesthesia. Firstly, the hip lesion was removed thoroughly and histopathologically examined to make a definitive diagnosis.

Different operation methods were selected for 29 patients according to different pathological types. Four patients younger than age 2 were treated with open reduction and external fixation by plaster hip spica. Acetabular reconstruction was performed for 25 patients. Among them, nine patients aged less than 6 with the AI < 40° and femoral head congruent with the acetabula underwent Salter osteotomy. Six patients aged 3–6 with the AI > 40°, femoral head not congruent with the acetabula and unclosed Y-shaped acetabular cartilages were treated with Pemberton's operation. In addition, Dega operation was used for seven patients aged 5–14 years with total hip dislocation. The hip shelf arthroplasty was performed for two patients aged more than 14 years with hip subluxation. One patient aged more than 14 with complete hip dislocation was treated via Chiari operation.

During the acetabular reconstruction, 16 patients underwent upper femoral rotational shortening (short, 1–3 cm; mean, 2 cm) osteotomies simultaneously. Six patients also underwent the femoral head and neck reconstruction, and their greater trochanter were moved down. Corrective osteotomy was performed in three patients to correct coax vara, and the neck–shaft angle was corrected to 25° (ranged, 15°–40°).

### Postoperative therapy

All affected limbs underwent external fixation postoperatively by plaster cast for 1–3 months. To prevent additional infection, cephalosporins were given for 3 days after surgery, whilst all patients were given antituberculosis therapy for 12–18 months. Postoperative X-ray photograph of each patient was taken. The exercise of patients was scheduled according to the stability of the hip joints and the healing of osteotomies.

## Results

Pathological examination indicated that all 29 cases were hip dislocation due to coxotuberculosis. Postoperative X-ray films showed well hip reduction of all patients. Postoperatively, 25 patients healed I incision surgery, while 4 patients were accompanied by skin antrum, which were cut, and the healing was delayed for 1.5 months (ranged, 1–3 months).

A total of 24 patients were followed up for 3 years (ranged, 2–5 years) (Table 2). No complication was detected, such as hip redislocation, pathologic fracture and looseness of internal fixation during the follow-up period. X-ray examination revealed that no dislocation reoccurred at 2 years after operation. The postoperative AI was 15°–20° in 22 patients and increased mildly to 25°–30° in 2 patients. The anteversion angle was 20° (ranged, 15°–20°) and the neck shaft angle was 125° (ranged, 110°–140°), indicating normal anatomical relation between the head and neck of hip (Figure 1). Among the patients associated with the femoral head and/or neck defect, 2 patients returned to normal femoral morphology, 17 patients showed malunion of femoral head, and 3 patients with femoral neck stump acted as femoral head presented a normal relationship of formal head and acetabula (Figure 2).

The article "Pathological dislocation of the hip due to coxotuberculosis in children: a 29-case report" was retracted in 2015. Reason: compromised peer review.

**Figure 1:** **Serial radiographs of a 6-year-old boy who presented with tuberculosis of left hip dislocation.** He was treated by left open reduction, Pemberton pelvis osteotomy, and corrective osteotomy in the left proximal femur. **(a)** Pre-operative. **(b)** Immediate post-operative. **(c)** 2 years post-operative.

**Figure 2:** **Serial radiographs of an 11-year-old girl who presented with tuberculosis of hip dislocation, thoracolumbar kyphosis, and spinal tuberculosis.** She was treated by right open reduction, Dega pelvis osteotomy, and subtrochanteric shortening osteotomy in the left proximal femur. **(a)** Pre-operative. **(b)** Immediate post-operative. **(c)** 2 years post-operative.

**Table 2:** Clinical outcome of 24 patients at 2 years after surgery

**Follow-up study**	**Patients**
Duration (years)	3 (ranged, 2–5)
Hip joint reduction	
Concentric reduction	21
Off-concentric reduction	3
Acetabular index	
15°–20°	22
25°–30°	2
Femoral morphology	
Normal	2
Malunion of femur head	17
Normal reduction of formal neck and acetabulum	3
Function of the hip joint	
Normal	8
Mild limitation of flexion and rotation	13
Fibrous ankylosis	3

The hip stability and weight-bearing were improved significantly. Hip pain was relieved. Twelve patients had residual mild lameness and four had moderate lameness, displaying leg length discrepancy (eight patients) with the average of 1.5 cm (ranged, 1–2 cm). After 2 years postoperatively, 8 patients had normal function of the hip joint; 13 cases had mild limitation of flexion and rotation, and 3 cases had fibrous ankylosis. The Harris hip score was 83 (ranged, 62–90).

## Discussion

Pathological dislocation of a joint is a complication that directly involves the joint surfaces, which is common in the hip joint. Destructive dislocation occurs commonly in tuberculosis of the hip because of a traveling acetabulum (destruction of the acetabulum) or in septic arthritis of the hip in infancy secondary to the total destruction of femur head. Distensile dislocation occurred because of rapid distension of the joint capsule due to effusion of synovial fluid or pus [7].

The article "Pathological dislocation of the hip due to coxotuberculosis in children: a 29-case report" was retracted in 2015. Reason: compromised peer review.

Since the pathologically dislocated hips generally did not become normal spontaneously during growth, detection at early stage was necessary and then appropriate remedial measures were performed [8,9]. If the abducted femoral head was hinged on the acetabular margin, which was common in subluxated and dislocated hips, spontaneous progressive cephalocotyloid improvement could not be expected without having a non-hinging hip by any measure. Johari et al. has reported the management of hip dislocations [10] and advocated a surgical intervention in failed closed reductions and in patients older than 2 years. In this study, we believed that patients even with active tuberculosis also needed aggressive treatment. The operation was performed after antitubercular chemotherapy for 2–4 weeks.

Davidson and Fernandez [11] have reported six cases of the dislocating type out of 31 cases of tuberculous hip (almost 20% incidence) in children younger than 14 years, and all 6 cases had poor outcomes. However, Campbell and Hoffman [12] have reported 13 cases of dislocating type of 74 hips (about 17% incidence), and the outcome was excellent/good in 46% of these cases (6 of 13). A poor outcome was found in those patients who had a narrow joint space after reduction. However, in the present study, all patients achieved satisfied outcomes which might be due to the different surgical procedures we adopted based on the age and the region, range, or extent of pathological dislocation.

Zadeh et al. [13] have reported the management of developmental hip dislocations and advocated that the age at operation might be a significant prognostic factor in the long follow-up, suggesting that 94% of patients under the age of 2 years achieved an acceptable outcome, while the proportion of patients aged 2–4 years and more than 4 years was 80% and 71%, respectively. Johari et al. [10] have reported a surgical intervention in failed closed reductions in patients older than 2 years and emphasized the need of supplemental procedures such as Dega osteotomy, Staheli shelf procedure, and femoral varus/derotational osteotomies combined with open reduction. Consistent with prior studies, in this study, patients under the age of 2 years were treated with open reduction associated with external fixation and the outcome was well.

Acetabular reconstruction is essential for patients with severe destruction of acetabulum and femoral head–neck as well as low stability of articular reduction. However, young age, the extent of coverage of the acetabular component by the graft, and secure fixation and mechanical loading of the graft might be impact factors [14,15]. Salter osteotomy was only fit for children aged 1–6 years with well-developed acetabular. Meanwhile, femoral head of these patients should be generally congruent with their acetabular roof. Salter osteotomy can provide a limited correction (15°–20°) which can be considered as a disadvantage in patients with severe dysplasia [16,17]. For children younger than 18 months, Salter osteotomy was contraindicated because satisfactory outcomes could be achieved by other measures [18]. Besides, the patients were usually too small to harvest or fix bone graft. For children older than 6 years, the prerequisites of complete reduction and reasonable congruity usually could not be met, hence it was contraindicated. Pemberton osteotomy was usually performed in patients aged 3–6 years with slightly shallower acetabulum and severe acetabular deficiency and was the most widely known incomplete transiliac osteotomy. Pemberton osteotomy starts approximately 10 to 15 mm above the anterior inferior iliac spine and curves gently posteriorly; the outer and inner tables of the ilium were osteotemized separately and ended at the level of the ilioischial limb of the triradiate cartilage halfway between the sciatic notch and the posterior part of the acetabular rim. Dega osteotomy was also a reshaping, incomplete osteotomy. The theoretical location of the hinge in the Dega osteotomy can involve, to varying degrees, the sciatic notch, the posterior portion of the inner pelvic cortex, the horizontal limb of the triradiate cartilage, and the symphysis pubis [19]. Similar to Pemberton osteotomy, Dega osteotomy also increases acetabular volume.

The article "Pathological dislocation of the hip due to coxotuberculosis in children: a 29-case report" was retracted in 2015. Reason: compromised peer review.

Subtrochanteric shortening osteotomy is a safe and predictable procedure to restore the anatomic hip center and trochanteric rotation without neurologic injury in high developmental hip dislocation [20]. It allows acetabular exposure, diaphyseal shortening, and facilitates femoral derotation. In this study, although the femoral head was nearly completely absent, the joint function of patients restored to an adequate level by placing stump of femur neck inside the acetabulum. For cases with coxa vara, derotational femoral shortening was performed combined with corrective osteotomy.

Many scholars have always disputed whether internal fixator could be left in the affected hip joint with pathological dislocation. Some researchers believe that using internal fixator will increase numerous of risk such as infection, recrudescence, foreign body reaction, and formation of fistula. We hold that the internal fixator should not be adopted in chronic inflammation infection period. Our clinical data indicated that using the limited internal fixation could greatly enhance the strength of acetabular bone after reconstruction. In addition, prompt removal of the internal fixator had not precluded wound from heal up. In the present study, we did not find any case that had complications caused by internal fixator.

The article "Pathological dislocation of the hip due to coxotuberculosis in children: a 29-case report" was retracted in 2015. Reason: compromised peer review.

## Conclusions

We have good results for surgical treatments in 29 patients with pathologic dislocation of tuberculous hip. Individualized surgical approach should be taken to treat tuberculosis hip in adolescent patients according to the pathological changes of affected acetabulum. In addition, based on this experience, the use of the early reconstructive surgery of the hip appeared effective even for patients with severely damaged acetabulum.

## Competing interests

The authors declare that they have no competing interests.

## Authors’ contributions

XJ and YL carried out the studies, participated in the sequence alignment, and drafted the manuscript. LL carried out the immunoassays with XY. MP participated in the sequence alignment. XY participated in the design of the study and performed the statistical analysis. DW conceived of the study, participated in its design and coordination, and helped to draft the manuscript. All authors read and approved the final manuscript.
